RETRACTED

# Status Quo of Occupational Identity of Nursing Staff in Rehabilitation Department and Its Relationship with Work Stressors

**DOI:** 10.1155/2022/9974311

**Published:** 2022-10-04

**Authors:** Ting Jiang, Qiaoli Jin

**Affiliations:** ^1^Rehabilitation Department, The First People's Hospital of Wenling, Wenling 317500, Zhejiang, China; ^2^General Practice, The First People's Hospital of Wenling, Wenling 317500, Zhejiang, China

## Abstract

Due to the continuous progress of social economy, medical and health technology and the development of disciplines have shown a trend of rapid development. In the current medical environment, quality nursing services are constantly promoted. Nursing staff are dedicated to their work to the best of their ability. Meanwhile, they should be rewarded with corresponding happiness and joy in their work. This study starts from the perspective of nursing management and psychology. On this basis, it investigates the occupational identity and work stress status of nursing staff. At the same time, the data are analyzed, and the relationship between occupational identity and work pressure is analyzed. This article provides a certain theoretical basis and support for the decision-making of relevant nursing managers, and also makes efforts to improve the professional identity and work happiness of nursing staff. In this study, which surveyed 596 rehabilitation nurses, the nurses' total occupational stress score was 74.52, with an average score of 2.12 points. The overall score for professional identity was 102.00, with an average score of 3.40 points. This belonged to the medium level. It showed that the occupational pressure of nurses should be paid attention to by relevant managers. Two of the five dimensions with the highest scores were occupational social support and occupational self-reflection. A negative correlation was found between occupational stress and its dimensions and occupational identity and its dimensions (*P* < 0.01).

## 1. Introduction

Nursing staff are on the clinical front line of caring for patients. Nursing staff have high occupational risks, high workload, fierce social competition, and fast-paced life, witnessing the pain of patients in their daily work, which has higher requirements on their physical, emotional, and spiritual aspects. Workplace stress is a globally recognized risk factor for employee health and safety. Nursing staff's repeated exposure to unpredictable challenges in nursing practice may cause them to experience symptoms of anxiety, exhaustion and stress, and excessive work stress. It not only affects their physical and mental health and aggravates work fatigue, but also affects the quality of work, which is not conducive to patient safety. In terms of teaching, it can provide theoretical support for the optimization of nursing professional personnel training programs for medical colleges and universities. In terms of medical treatment, it can provide a reference for managers to reduce the work pressure of nursing staff and strengthen the management of nursing deficiency. This study explores the root causes of nursing deficits from the perspective of work stress and understands the mechanism of occupational identity. This not only helps managers to formulate countermeasures to reduce the impact of nursing staff's work pressure on nursing deficiency and helps nursing managers to pay attention to the positive impact of professional identity, but also helps stabilize the nursing talent team and reduce nursing deficiency. It is hoped that through this study, the stress status of nursing staff can be better understood, and the relationship between work stress and occupational identity and nursing deficiency can be explored, thus attracting the attention of hospitals and medical colleges, and reducing the work pressure of nursing staff, so as to improve their professional identity and strengthen professional emotion as well as stabilize the nursing team. At the same time, the study of nursing deficiency in this study has certain practical significance for promoting the recovery of patients.

RETRACTED

Stress resilience is a trait and skill that caregivers can develop. Leng's research examined the current status and influencing factors of nursing staff's ability to cope with stress, as well as the work stress felt by nursing staff. Studies have found that nursing staff's ability to withstand stress is significantly related to age, working years, clinical grade, and education level [1]. Emishaw assessed nursing staff's job stress and identifies factors that contribute to stress. Using a mixed-site, cross-sectional approach, a detailed survey of nursing staff perceptions was conducted, with trained nursing staff involved in the data collection process and supervision [2]. Stress factors at work in the NICU can outweigh satisfaction factors, leading to job dissatisfaction and turnover. Fiske surveyed current NICU stressors, satisfaction, and coping processes, and analyzed open-ended responses through iterative coding and topic clustering. As a result, most nursing staff felt that nursing in the intensive care unit was stressful [3]. Unresolved work stress can lead to burnout, compassion fatigue, and disengagement. Research by Klein found that occupational stress can also have a negative impact on organizations. A quantitative online cross-sectional survey of nursing staff was conducted, including open-ended questions about work stress and balancing work and family life [4]. Evidence and research showed that nursing is one of the most stressful jobs. Dolatshad's study found the impact of occupational stress on employees' mental health. Feelings of mental health are widely influenced by an individual's perceptions of events and occupational stressors. Stress reduces people's attention, concentration, decision-making ability, and judgment, which is inversely related to the quality of care [5]. However, research on job stressors for nursing staff has not been linked to other studies.

RETRACTED

Research by Frechette found that professional identity can improve nursing staff retention and quality of care. This study was conducted using an explanatory phenomenological design, with data collection through face-to-face interviews, photographs, participant observations, and document review [6]. Paramedic occupational self-concept is related to how individuals see themselves as professionals, while nursing work is related to how paramedics see themselves. The purpose of Kusnanto's study was to establish a professional self-perception model of nursing staff productivity, using an interpretive crossover design. It was found that there is also a relationship between professional nursing staff's self-perception, which may improve nursing staff's productivity [7]. Yang found that there were few studies on the degree of embarrassment and the factors related to embarrassment among nursing staff through research. He also used logistic regression to study the factors related to the level of shame [8]. Although the occupational identity of NPs is important in determining the characteristics of nursing practice, few studies have examined the occupational identity of NPs that overlap with immigration experiences. Seo's research findings analyzed the data using content analytics. The results indicated that their participants' focus on listening, interpersonal relationships, and patient care education would develop new roles in nursing [9]. Little was known about how the education and professional certification of critical care paramedics affects patient outcomes. Gigli studied not only the educational level and professional certification of ICU nursing staff, but also their professional identity, self-efficacy, and role clarity and their relationship [10]. However, these studies did not link the status of occupational identity and work stressors.

## 2. Deconstruction Methods on the Relationship between Stress and Professional Identity

### 2.1. Development Trend of Stress and Professional Identity of Nursing Staff

Nursing workers are an indispensable strong force in the medical industry. With the aging of the Chinese population, the demand for nursing workers is increasing [11]. In the current medical environment, it is particularly important to pay attention to the pressure in the work of nursing staff and the degree of identification with their own profession [12]. Lack of care has become a global concern, affecting patient safety and quality of care, and severely hindering patient treatment and recovery, which contributes to poor nursing staff and patient outcomes. Research on nursing deficits in China started relatively late [13]. The model of stressor-stress experience-stress outcome is shown in Figure 1.

RETRACTED

As shown in Figure 1, potential stressors include environmental, organizational, and personal factors. Stressful experiences are the result of a combination of underlying stressors and individual differences. Individual differences include personal cognition and social support. Different from external factors of work, it mainly uses internal factors of individual differences to explain the reasons why work pressure varies from person to person, and then produces different physiological, psychological, and behavioral symptoms and other stress results [14]. Whether potential stressors can be transformed into actual stress mainly depends on differences in personality characteristics and individual coping. Coping style, also known as coping strategy, is a way for individuals to deal with stress and maintain psychological balance under pressure. It is continuous and dynamic and can be divided into positive coping and negative coping. Individual characteristics and coping styles are different, resulting in different stress outcomes. In this study, the stressors of nursing staff focus on work stressors, coupled with different general demographic data such as work department and gender, and use occupational identity as a mediating variable to explore individual differences in nursing staff stress [15]. Occupational recognition can be understood as the personal recognition of the nursing profession by nursing staff, indicating that they are willing to overcome all difficulties and obstacles in order to realize their own life and social value. It acts as an intrinsic driver that affects the way caregivers respond to stress, resulting in a different stress outcome, that is, nursing loss.

### 2.2. Application of Neural Network in Emotion and Stress Recognition

Traditional machine learning algorithms usually have problems with relatively simple mathematical expressions, which cannot accurately describe the characteristics of features. Therefore, the neural network algorithm based on multilayer perceptron has received extensive attention from researchers [16]. Neural networks have also shown excellent performance in areas related to emotion and stress recognition [17, 18]. Therefore, some researchers chose to convert the filtered data into a picture or sequence format, and directly input it into the neural network. The feature extraction, feature transformation, and recognition of the data are done by the network. The framework of the stress recognition algorithm based on convolutional neural network is shown in Figure 2.

RETRACTED

As shown in Figure 2, the neural network itself has the ability to extract features. For example, in the convolutional neural network, the process of processing the original image by the convolution kernel is essentially a process of performing matrix operations on tensors through learnable filters to obtain feature maps of different scales and values [19–22]. Based on this thought, a common physiological signal emotion recognition algorithm flow is shown in Figure 3.

As shown in Figure 3, the use of the neural network to extract and identify the features of the original signal can effectively extract all kinds of information contained in the signal, but it also has certain shortcomings [23]. Since the signal sampling frequency of the original signal is usually high and the amount of signal data is large, the design requirements for the network structure are high. If the network is too large and too deep, the amount of parameters is too large, which is difficult to train and prone to overfitting. If the network is too small and too shallow, the information contained in the signal cannot be fully extracted [24].

### 2.3. Frequency Domain Characteristics of Pulse Signals

Short-time Fourier transform is often unable to cope with various physiological signals with complex distribution, while wavelet transform is widely used in the analysis of nonstationary physiological signals due to its variable window length [25]. For discrete time series, the wavelet transform is essentially multilevel frequency domain segmentation, as shown in the following formula:

(1) $$\begin{array}{c} DWT\left(i,j\right)=\overset{+\infty }{\underset{-\infty }{\int }}f\left(k\right)\times \frac{1}{\sqrt{2i}}\alpha \left(\frac{k-2ij}{2i}\right)dk\text{.} \end{array}$$

The essence of discrete wavelet transform is to divide the signal into a high-frequency details coefficient (cD) and a low-frequency approximation coefficient (cA) through high- and low-frequency filters, further decomposing the approximate components until the number of decomposition layers reaches the wavelet transform to the set number of layers.

The frequency domain feature used in this article is the proportion of the frequency band energy of each layer in the total energy after wavelet transform, and its mathematical expression is as follows:

(1) The in-band energy of a certain layer is calculated as shown in the following formula based on Pascal's theorem:
  (2) $$\begin{array}{c} Energy=\overset{M}{\underset{m=1}{\sum }}s_{m}^{2}\text{.} \end{array}$$
(2) For the frequency band energy ratio, the calculation is performed as follows:
  (3) $$\begin{array}{c} {Ratio\_Energy}_{i}=\frac{{Energy}_{i}}{\overset{N}{\underset{j=1}{\sum }}{Energy}_{i}}\text{.} \end{array}$$

For the discriminator *D*, D wants to identify as accurately as possible whether the input is from the generative network *G* or the real data, that is to maximize the expression, as shown in the following formula:

(4) $$\begin{array}{c} \max_{D}\left(\overset{\alpha ∼\overset{da\;ta}{p}\left(\alpha \right)}{E}\left[\log\;D\left(\alpha \right)\right]\right.\text{.} \end{array}$$

For the generator *G*, G hopes to generate data that cannot be accurately distinguished as “real” by *D* through training. That is, through training, the objective function shown in the following formula can be minimized:

(5) $$\begin{array}{c} \min_{G}\underset{D}{\max\;V\left(G,D\right)=}\left(\overset{\alpha ∼\overset{da\;ta}{p}\left(\alpha \right)}{E}\left[\log\;D\left(\alpha \right)\right]\right.\text{.} \end{array}$$

The training of GAN is carried out in stages, because *G* and *D* need to be trained separately to be optimal. Therefore, the parameter update formula based on gradient ascent for the discriminator *D* is shown in the following formula:

(6) $$\begin{array}{c} \nabla_{\theta_{g}}\frac{1}{n}\sum_{j=1}^{n}\left[\;\log\;D\left(\underset{n}{\alpha }\right)\right.+\log\left(1-D\left.\left(\underset{n}{\alpha }\text{)}\right)\right]\right. \end{array}$$

After *k* times of training, the discriminator *D* is fixed, and the parameter update formula based on gradient descent is applied to the generator *G*, as shown in the following formula:

(7) $$\begin{array}{c} \nabla_{\theta_{g}}\frac{1}{n}\sum_{j=1}^{n}\log\left(1-D\left.\left(\underset{n}{\alpha }\right)\right]\right. \end{array}$$

If the value of *k* is too large, the update of *D* will be too frequent, which will lead to serious gradient disappearance in the training of *G*.

RETRACTED

Therefore, after GAN was proposed, a large number of researchers optimized the native model of GAN. The optimized model has been applied to solve various problems that are difficult to solve by traditional neural networks. Among them, the design concepts of adversarial networks and discriminators have been deeply developed and improved. They have been used by some researchers to optimize interference information in recognition problems.

### 2.4. Optimization of Decision Tree Algorithm by Association Rules

Most existing decision tree algorithms focus on feature selection metrics or improved pruning algorithms. The number of relevant rules extracted by many relevant rule extraction algorithms is always surprisingly large without any contribution to the extraction result. In order to build new features through association rules, it is important to know which rules to use.

In the approximate exact rule algorithm, a set of rules are generated and the previous rule elements are combined with new features and added to the original dataset.

The value of the new attribute ABR_1_ is shown as follows:

(8) $$\begin{array}{c} {ABR}_{1}=\left\{\begin{array}{cc} 1\text{,} & if,X_{1}=a_{11},X_{2}=a_{31},X_{3}=a_{31}\\ 0\text{,} & else \end{array}\right) \end{array}$$

First, the candidate ABR_*i*_ feature to be evaluated is the root node of the decision tree. The information content of the root node is shown as follows:

(9) $$\begin{array}{c} G_{root}=-\overset{m}{\underset{j=1}{\sum }}\frac{m_{j}}{M}{\mathrm{Log}}_{2}\frac{m_{j}}{M} \end{array}$$

where *m* represents the total number of records in the sample dataset and *m*_*j*_ is the number of the jth value of the ranking attribute.

If the sample data are classified and evaluated by ABR_i_ attribute, the number of data records for = ABR_*i*_1 attribute is *M*_1_, as shown in the following formula:

(10) $$\begin{array}{c} M_{1}=M*\frac{sup\left(R_{i}\right)}{conf\left(R_{i}\right)}\text{.} \end{array}$$

In the data record of attribute *ABR*_*i*_ = 1, the number of records of category attribute *B*=*b*_*i*_ is *N*_2_, as shown in the following formula:

(11) $$\begin{array}{c} M_{2}=M*sup\left(R_{i}\right) \end{array}$$

On the other hand, a record with *a* = ABR_*i*_1 attribute has an unknown number of B-type attribute values of *b*_*i*_. The amount of information contained in this type of data is ignored here, since exact approximation algorithms are used to generate exact approximation rules. Therefore, the amount of information contained in the records of the dataset matching = ABR_*i*_1 is shown in the following formula:

(12) $$\begin{array}{c} G_{1}=\frac{M_{1}}{M}\left[-\frac{M_{2}}{M_{1}}{\mathrm{Log}}_{2}\frac{M_{2}}{M_{1}}\right]\text{.} \end{array}$$

### 2.5. C4.5 Algorithm

In the decision tree algorithm C4.5, the test condition for feature selection in the decision tree model is the information gain rate. It represents the amount of categorical information required for a given data sample, as shown in the following formula:

(13) $$\begin{array}{c} Info\left(D\right)=-\overset{m}{\underset{i=1}{\sum }}p_{i}\log_{2}\left(p_{i}\right) \end{array}$$

where *p*_*i*_ is the proportion of *C*_*i*_ in the sample, which can generally be calculated by *C*_*i*_/*d*.

RETRACTED

Based on the information gain, the information gain rate is formulated. SplitInfoA (*D*) is an entropy concept when the value of attribute A is used as the basis for sample splitting, as shown in the following formula:

(14) $$\begin{array}{c} {SplitInfo}_{A}\left(D\right)=-\overset{v}{\underset{j=1}{\sum }}p_{j}\log_{2}p_{j}\text{.} \end{array}$$

where *p*_*j*_ is the proportion of the sample with the same value *a*_*j*_ on A, which can generally be calculated by *d*_*j*_/*d*. Finally, the formula of the information gain rate of attribute A to divide the dataset is obtained, as follows:

(15) $$\begin{array}{c} GainRatio\left(A\right)=\frac{Info\left(D\right)-{Info}_{A}\left(D\right)}{SplitInfo_{A}\left(D\right)} \end{array}$$

The specific calculation formula used by the C4.5 algorithm is shown in the following formula:

(16) $$\begin{array}{c} GainRatio\left(A\right)=\frac{Gain\left(A\right)}{SplitInfo_{A}\left(D\right)}\text{.} \end{array}$$

### 2.6. Loss Function Design

This article uses the WESAD dataset and the SCUT dataset to verify the model experimentally. This paper includes two classifications and three classifications. The three-category labels are neutral, stress, and pleasure. The two-category labels are stress and stress-free (combining neutral and pleasant).

It can be seen from the schematic diagram of the network structure that two classifiers participate in training at the same time. Therefore, the loss function of the training process consists of three parts.

In this article, the focal loss function is used in the three-category/two-category problem to solve the problem of class imbalance. The loss function of the pressure classification part is shown in the following formula:

(17) $$\begin{array}{c} \overset{stress}{Loss}=\overset{3}{\underset{x=1}{\sum }}-\delta_{t}{\left(1-\phi_{x}\right)}^{\gamma }\;\log\left(\phi_{x}\right) \end{array}$$

Considering that the number of samples of each person is roughly the same and does not require special processing for balancing, this article chooses the cross-entropy function as the identity classification function, and the calculation formula is shown in the following formula:

(18) $$\begin{array}{c} \overset{i\;de\;ntify}{Loss}=-\frac{1}{M}\overset{M-1}{\underset{j=0}{\sum }}\overset{M-1}{\underset{j=0}{\sum }}\overset{j,k}{x}\log\phi_{j,k}\text{ .} \end{array}$$

Combining the above various loss functions, it is necessary to use different coefficients to make each loss function similar in magnitude to prevent the training process from being biased. Therefore, the overall loss function is shown in the following formula:

(19) $$\begin{array}{c} Loss_{mo\;de\;l}=Loss_{stress}+\overset{1}{\lambda }Loss_{reg}+\overset{1}{\lambda }Loss_{i\;de\;ntify} \end{array}$$

RETRACTED

## 3. Relationship between Occupational Identity and Work Stressors of Nursing Staff

### 3.1. Investigation Method

This study used a cross-sectional study and convenience sampling method. The survey method was a questionnaire survey. There were two ways to conduct this survey. The first way was to distribute them uniformly to research subjects by trained investigators. After the investigator stated the research purpose, the research subjects participated voluntarily, filled in anonymously, and took it back on the spot. The whole process took about 30 minutes, and the valid questionnaire was returned after filling out. The second way was to distribute the online software to the research subjects by the person in charge, and valid questionnaires were collected after online submission. Before the questionnaire survey, a research group has been established, and the questionnaire survey was completed by the staff of the research group.

### 3.2. Logical Relationship

On the basis of surveying the general data, firstly the occupational identity and work pressure were investigated, respectively, and the univariate analysis and multivariate analysis were completed, and then carry out the correlation analysis between occupational identity and work pressure. Univariate and multivariate analyses were performed. Then, the correlation analysis between occupational identity and job stress was carried out. Finally, the corresponding conclusions and results were drawn and analyzed. The pre-investigation has been completed in our hospital before the formal investigation, which ensured the accuracy and scientificity of the results.

### 3.3. Quality Control

This study was sampled according to the inclusion and exclusion criteria. Before distributing the questionnaires, the hospital leaders were contacted. After obtaining their approval, the researchers then contacted the department head nurses on a case-by-case basis. After asking for their consent, the significance of the research, matters needed attention, etc. were explained to them. It was indicated that the personal name was not required to be written on the questionnaire, and the obtained data were only used as the information of this research, which would not be leaked so that the nursing staff could fill in the truth. After the questionnaires were distributed, the time when the questionnaires would be returned was agreed. During this period, the head of the nursing staff or the person in charge of the department needed to be communicated with from time to time. After the questionnaires were collected uniformly, the researchers repeatedly reviewed the completeness and logic of the questionnaires one by one, and then unified coding after eliminating invalid questionnaires. Data entry was performed using Exce12016. After recording, the accuracy of the entry was checked. Specifically, all variables entered were analyzed using SPSS 21.0 line frequency. If there are missing values and answering logic confusion, they should be supplemented and corrected in time. Finally, all data were checked against the original data.

RETRACTED

### 3.4. Basic Information of Nursing Staff

A total of 596 nursing staff were surveyed in this study. Among the departments, surgical nursing staff accounted for the largest proportion, accounting for 48.7% of the total number of nursing staff. The number of women was much higher than that of men, accounting for 97.3%. The age range was from 21 to 55 years, with the most nursing staff in the age group of 25 to 34 years, accounting for 58.7%. Some basic information is shown in Table 1.

As shown in Table 1, the remaining statistical bases are represented by text. In marital status, the number of married nursing staff was more than that of unmarried, accounting for 66.1% of the total number of nursing staff. Among the number of children, the proportion of nursing staff with one child was the highest, which was 46.0%. Among the educational level, undergraduates accounted for the highest proportion, with a rate of 65.4%, followed by junior colleges with 31.9%. Secondary school nursing staff was only 2.3%. Among the professional titles, nurses accounted for the highest proportion, 47.3%, followed by 24.2% of nursing staff. Nursing staff with 2 to 4 years of working experience accounted for the highest proportion, with a rate of 35.7%. The average monthly income was mainly concentrated in 4001–8000 yuan, accounting for 71.1% of the total number of nursing staff. Nursing staff with an average weekly working time of 41–50 hours accounted for the largest proportion, accounting for 66.1%. Nursing staff with an average of 0.1 to 0.5 hours of delayed get off work per day were the most, accounting for 52.9% of the total. Nursing staff who were often in charge of more than 12 patients accounted for the most, accounting for 33.1%. The proportion of nursing staff who believed that the nursing staff was adequate was basically the same as the proportion of nursing staff who believed that the nursing staff was insufficient. Nursing staff who thought that the working environment of the department was good accounted for the most, accounting for 50.2%, followed by 41.1% who thought that the working environment of the department was normal. Nurses who got on well with colleagues far outnumbered those who did not. There were more nursing staff with night shifts than without night shifts.

RETRACTED

## 4. Nursing Relationship Results and Deconstruction

### 4.1. Overall Characteristics of Work Stress of Nursing Staff

Nursing staff work stress and dimension scores are shown in Figure 4.

As shown in Figure 4, the total score of work stress of nursing staff in this study was 74.52 points, with an average score of 2.12 points. The mean scores for the five dimensions of work-related stress among nurses were, in order, time allocation and workload, professional and work-related aspects of nursing, patient care, working environment and tools, and management and interpersonal relationships.

### 4.2. Differences in Work Stress among Nurses with Different Demographic Characteristics

After analysis, the work stress score of nursing staff was reflected in different departments, gender, age, working hours per week, the number of hours delayed from getting off work every day, and the number of patients in charge. Figures 5 and 6 show a comparison of differences in work stress among nursing staff across different demographic characteristics.

As shown in Figures 5 and 6, after a pairwise comparison, the work pressure of nursing staff aged ≤24 years was lower than that of nursing staff of other age groups. Married caregivers were more stressed than unmarried. Nursing staff with children were more stressed than those without children. The pressure of nurses with the title of nurses and nurses in charge was higher than that of nurses, and the pressure of nurses in charge was higher than that of nurses. Nursing staff who worked for 5–9 years and ≥10 years had higher stress than those who worked for 2–4 years. Nurses working >60 hours a week were more stressed than those working other hours. Nursing staff who left work late each day were more stressed than those who did not leave work late.

There were differences in job stress scores among nursing staff with different demographic characteristics. Nursing staff aged ≤24 years had lower work pressure than those of other age groups. The job title of nursing staff was less stressful than that of nurses and nurses in charge. The analysis showed that nursing staff of this age group had just entered the workplace, who were less affected by external factors and were more likely to self-regulate. Married caregivers in the survey were more stressed than unmarried ones. Caregivers with children were more stressed than those without children. It reflected that nursing staff were greatly influenced by family factors when they faced work pressure. Nursing staff who worked for 5–9 years and ≥10 years had higher stress than those who worked for 2–4 years. It might be because nursing staff with long working years often lost the freshness of daily work and were mostly responsible for department management, education, and scientific research. Nursing managers needed to be prompted to pay attention to their psychological state, provide emotional support, and reasonably allocate workload. The stress of nursing staff who worked >60 hours per week was higher than those who worked ≤40 hours, 41–50 hours, and 51–60 hours. The working pressure of the nursing staff who delayed leaving work for 0.1–0.5 h, 0.6–1 h, and >1 h per day was higher than that of the nursing staff who did not leave work late. Nursing staff were more likely to feel fatigued if they worked longer or the number of patients they were in charge of was larger. They worried about making mistakes in their nursing work, thereby increasing the psychological burden. Under-staffed caregivers were more stressful than fully staffed. The working pressure of nurses with an average or poor working environment in the department was higher than those with a good working environment. Nursing staff with a poor working environment were also more stressed than those with a normal working environment. It showed that the better the working environment of the department, the less the working pressure of the nursing staff, which reflected the importance of the staffing of hospital nursing staff and the working environment.

RETRACTED

### 4.3. Overall Characteristics of Nursing Staff's Professional Identity

The occupational identity and dimension scores of nursing staff are shown in Figure 7.

As shown in Figure 7, the total score of the professional identity of the nursing staff in this study was 102.00 points, with an average score of 3.40 points. The average scores of the five dimensions of nurses' occupational identity were occupational social support, occupational self-reflection, occupational frustration management, occupational cognitive evaluation, and occupational social skills.

### 4.4. Differences in Occupational Identity among Nurses with Different Demographic Characteristics

Figures 8 and 9 show a comparison of differences in occupational identity among nurses with different demographic characteristics.

As shown in Figures 8 and 9, after a pairwise comparison, the occupational identity scores of the obstetrics and ICU nurses were higher than those of the internal medicine nurses. Nursing staff aged ≤24 and ≥ 45 years scored higher than those aged 35–44 years. Unmarried caregivers scored higher than those who were married. Caregivers without children scored higher than those with one child. In terms of professional titles, the scores of professional identity of nursing staff are higher than those of nurses and nurses in charge. Nurses with 2 to 4 years of work experience higher scored than those with ≥10 years of experience. Nurses who did not leave work late each day scored higher than those who were late. Nursing staff with ≤6 and 7–8 patients who were often responsible for the number of patients scored higher than those with >12 patients. In terms of staffing of nursing staff, adequate nursing staff scored higher than those with insufficient staffing. Nursing staff with a good working environment in the department scored higher than those with a normal and a poor working environment.

RETRACTED

### 4.5. Multivariate Deconstruction of Factors Influencing the Occupational Identity of Nursing Staff

This survey used occupational identity as a dependent variable. Single factors such as years of work, job title, marriage, and child scores were used as independent variables. Then, after performing multiple linear regression analysis, the multivariate analysis of factors affecting the occupational identity of nursing staff is shown in Table 2.

As shown in Table 2, a univariate analysis was performed on the factors affecting nurses' professional identity. The results showed that there were statistically significant differences in the scores of seniority, professional title, marriage, and children (*P* < 0.05). Length of service (6–10 years), job title (nursing staff), marriage (married), and children (one child) are factors of occupational identity. The results of multiple linear regression analysis showed that working years, professional title, marriage, and children were the main factors affecting nurses' professional identity (*P* < 0.05).

The relationship between work stress and professional identity of nursing staff is shown in Table 3.

From the results in Table 3, it can be seen that there was a negative correlation between nursing staff's work stress and its various dimensions and occupational identity and its various dimensions (*P* < 0.01). In addition, occupational social skills scored the lowest in this study. This may be related to the scheduling of nursing staff. Nursing staff are busy with their daily work, with less time at their disposal, and have less social and recreational activities. In addition to family members, the people who have the most contact with nursing staff are patients and their families. At present, the relationship between doctors and patients and nurses is tense. Nursing staff are cautious in their work and pay less attention to social skills than nursing knowledge and skills.

RETRACTED

There were differences in the occupational identity scores of nursing staff with different demographic characteristics. Both obstetrics and ICU nursing staff had higher occupational identity scores than medical nursing staff. This is slightly different from previous studies possibly because of a different sample source. Nurses aged 35–44 years scored lower than those aged ≤24 and ≥ 45 years. It might be because the subject in this survey was a tertiary first-class general hospital, and the nursing staff of this age group had to not only face the pressure of family, but also face the pressure of hospital assessment and self-development. If they do not handle it properly, they are prone to burnout, leading to a low level of professional identity. Nurses who did not leave work late each day scored higher than those who were late. Nursing staff with ≤6 and 7–8 patients who were often responsible for the number of patients scored higher than those with >12 patients. Nursing staff who left work late every day and were responsible for a large number of patients were prone to burnout in nursing work and experience less sense of value in their work.

## 5. Conclusions

In this study, the total score of nursing staff's work stress was 74.52 points, and the average score was 2.12 points, which belonged to the middle level. It showed that the work pressure of nursing staff needs to be paid attention to by relevant managers. Five dimensions scored higher. The time allocation and workload dimensions were 2.41 points, and the nursing and work dimensions were 2.28 points. Two of the highest scores on these five dimensions were professional social support and professional self-reflection, which might be due to patients, their families, and colleagues being more supportive of the work of caregivers. The support of patients, families, and colleagues played a pivotal role in the professional identity of nursing staff. This support not only enhances the well-being and values of caregivers, but also makes them more cherished and engaged in care work, effectively relieving their work stress, which reduces burnout and encourages caregivers to remain relaxed and positive at work. The research showed that nursing staff had moderate levels of job stress and a moderate sense of professional identity. The higher the occupational stress of nursing staff is, the lower the occupational identity level of nursing staff will be. This study only conducted a cross-sectional survey of nurses, and did not conduct qualitative research and intervention research, which can be carried out in the future to make the results and conclusions more convincing.

RETRACTED

## Figures and Tables

**Figure 1:** Stressor-stress experience-stress outcome model.

**Figure 2:** Framework diagram of the stress recognition algorithm based on convolutional neural network.

**Figure 3:** Algorithmic framework for classifying raw signals using neural networks.

**Figure 4:** Nursing staff work stress and dimension scores.

**Figure 5:** Comparison of differences in work pressure in departments and age distribution characteristics of nursing staff. (a) Department. (b) Age.

**Figure 6:** Comparison of differences in work stress on the characteristics of weekly working hours and daily delayed hours for nursing staff. (a) Hours of work per week. (b) Hours delayed from getting off work per day.

**Figure 7:** Occupational identity and dimension scores of nursing staff.

**Figure 8:** Comparison of differences in occupational identity among nursing staff in terms of department and age distribution characteristics. (a) Department. (b) Age.

**Figure 9:** Comparison of differences in occupational identity among nursing staff on the characteristics of working hours per week and hours delayed from getting off work per day. (a) Hours of work per week. (b) Hours delayed from getting off work per day.

**Table 1:** Basic demographics of nursing staff (*N* = 596).

Project	Grouping	Number of people	Composition ratio (%)
Department	Internal medicine	220	36.9
	Surgical	290	48.7
	Obstetrics and gynecology	59	9.9
	Pediatrics	14	2.3
	ICU	13	2.2
Gender	Male	16	2.7
	Female	580	97.3
Age	≤24 years old	93	15.6
	25∼34 years old	350	58.7
	35∼44 years old	107	18.0
	≥45 years old	46	7.7

**Table 2:** Multivariate analysis of factors influencing the occupational identity of nursing staff.

Influencing factors	Nonstandard regression coefficients		Standard regression coefficients	t	*p*
	*β*	SE			
Constant term	0.340	0.183	—	1.860	0.064
Working years	0.217	0.048	0.306	4.496	<0.001
Job title	−0.183	0.032	−0.345	−5.646	<0.001
Marriage	−0.328	0.040	−0.501	−8.138	<0.001
Child	00.429	0.023	1.128	18.849	<0.001

**Table 3:** Correlation between work stress and occupational identity of nursing staff.

	Professional identity	Cognitive evaluation	Social support	Social skills	Coping with setbacks	Self-reflection
Nursing	−0.355	−0.267	−0.272	−0.292	−0.264	−0.321
Time workload distribution	−0.426	−0.297	−0.340	−0.305	−0.257	−0.368
Working environment	−0.305	−0.241	−0.211	−0.262	−0.213	−0.274
Patient care	−0.354	−0.282	−0.307	−0.290	−0.233	−0.327
Interpersonal relationship	−0.314	−0.331	−0.235	−0.348	−0.285	−0.326
Work pressure	−0.437	−0.357	−0.345	−0.376	−0.314	−0.405

RETRACTED

## Data Availability

Data sharing is not applicable to this article as no datasets were generated or analyzed during this study.
